The article "Molecular Mechanisms of Nanosized Titanium Dioxide–Induced Pulmonary Injury in Mice" was retracted in 2024. Reasons: unreliable results or conclusions; concerns about the data; concerns about the results or conclusions; concerns about the citations.

# Molecular Mechanisms of Nanosized Titanium Dioxide–Induced Pulmonary Injury in Mice

**DOI:** 10.1371/journal.pone.0055563

**Published:** 2013-02-07

**Authors:** Bing Li, Yuguan Ze, Qingqing Sun, Ting Zhang, Xuezi Sang, Yaling Cui, Xiaochun Wang, Suxin Gui, Danlin Tan, Min Zhu, Xiaoyang Zhao, Lei Sheng, Ling Wang, Fashui Hong, Meng Tang

**Affiliations:** 1 Medical College of Soochow University, Suzhou, China; 2 Key Laboratory of Environmental Medicine and Engineering, Ministry of Education, School of Public Health, Southeast University, Nanjing, China; 3 Jiangsu key Laboratory for Biomaterials and Devices, Southeast University, Nanjing, China; University of North Dakota, United States of America

## Abstract

The pulmonary damage induced by nanosized titanium dioxide (nano-TiO_2_) is of great concern, but the mechanism of how this damage may be incurred has yet to be elucidated. Here, we examined how multiple genes may be affected by nano-TiO_2_ exposure to contribute to the observed damage. The results suggest that long-term exposure to nano-TiO_2_ led to significant increases in inflammatory cells, and levels of lactate dehydrogenase, alkaline phosphate, and total protein, and promoted production of reactive oxygen species and peroxidation of lipid, protein and DNA in mouse lung tissue. We also observed nano-TiO_2_ deposition in lung tissue via light and confocal Raman microscopy, which in turn led to severe pulmonary inflammation and pneumonocytic apoptosis in mice. Specifically, microarray analysis showed significant alterations in the expression of 847 genes in the nano-TiO_2_-exposed lung tissues. Of 521 genes with known functions, 361 were up-regulated and 160 down-regulated, which were associated with the immune/inflammatory responses, apoptosis, oxidative stress, the cell cycle, stress responses, cell proliferation, the cytoskeleton, signal transduction, and metabolic processes. Therefore, the application of nano-TiO_2_ should be carried out cautiously, especially in humans.

## Introduction

Nanosized titanium dioxide (nano-TiO_2_) particles, due to their high surface area to particle mass ratio, have been increasingly used as catalysts and are now being commercially manufactured for use in medical, diagnostic, energy, component, and cosmetic applications as opposed to bulk TiO_2_ (micrometer-sized) [1], [2]. However, concerns have been raised over the safety of nano-TiO_2_ particles, as the toxicological effects of nano-TiO_2_ have been demonstrated through several exposure routes, including dermal, oral, and pulmonary. Especially, following inhalation, nano-TiO_2_ particles are internalized by clathrin-mediated endocytosis, caveolin-mediated endocytosis, and macropinocytosis by both phagocytic and non-phagocytic cells [3]. Reportedly, industrial nano-TiO_2_ production, which includes a process that produces heavy nano-TiO_2_ dust, increased the risk of pneumoconiosis to workers. Several reports have shown that human exposure to nano-TiO_2_ occurs through different pathways, including inhalation and exposure of the integumentary system. The pulmonary responses induced by inhaled nanoparticles (NPs) are considered to be greater than those produced by micron-sized particles because of the increased surface area to particle mass ratio [4], [5]. In vitro studies have demonstrated that both rutile and anatase nano-TiO_2_ impaired cellular function of human dermal fibroblasts and decreased cellular area, proliferation, mobility, and ability to contract collagen, with the latter being more potent in inducing damage [6]. Animal experiments arrived at the same results regarding the relationship between nano-TiO_2_ exposure and lung inflammation. Moreover, inhaled NPs, after deposition in the lungs, largely escaped the alveolar macrophage surveillance system and gained greater access to the pulmonary interstitium by translocation from alveolar spaces through the epithelium [7]. Liu et al. [8] reported that intratracheal administration of nano-TiO_2_ (5 nm) led to significant increases in lactate dehydrogenase (LDH) and alkaline phosphatase (ALP) activities, infiltration of inflammatory cells, and interstitial thickening in the rat lung.

Our previous in vivo studies demonstrated that exposure to nano-TiO_2_ induced pulmonary inflammation and apoptosis in mice, which were associated with expression levels of nuclear factor–κB, tumor necrosis factor-α, cyclooxygenase-2, nuclear factor erythroid 2-related factor 2, heme oxygenase 1, glutamate-cysteine ligase catalytic subunit, interleukin (IL)-2, -4, -6, -8, -10, -18, and -1β, cytochrome P450 1A1, NF-κB-inhibiting factor, and heat shock protein 70 in the mouse lung [9], [10]. Although the above-mentioned studies clarified the toxicological effects of nano-TiO_2_, further studies are needed to elucidate the synergistic molecular mechanisms of multiple genes activated by nano-TiO_2_-induced pulmonary inflammation and apoptosis in animals and humans.

DNA microarrays have been used to identify gene clusters involved in the progression of pulmonary fibrosis and lung injury [11]–[14]. Furthermore, gene expression profiling has been performed to elucidate the toxicological effects of single-walled carbon nanotubes, nano-TiO_2_, and C_60_ fullerene particles [15]–[17]. In the present study, we investigated gene expression profiles of the murine lung to explore mechanisms of immune/inflammation responses, apoptosis, and oxidative stress induced by exposure to nano-TiO_2_ for 90 consecutive days to serve as a reference for future mechanistic studies on the effects of nano-TiO_2_ and other NPs in pulmonary toxicity to animals and humans.

## Materials and Methods

### Preparation and Characterization of TiO_2_ NPs

Nanoparticulated anatase TiO_2_ was prepared via controlled hydrolysis of titanium tetrabutoxide. The details of the synthesis and characterization of nano-TiO_2_ have been previously described by our group [18], [19]. TiO_2_ powder was dispersed on the surface of 0.5% (w/v) hydroxypropyl methylcellulose (HPMC) K4M solution, treated ultrasonically for 15–20 min, and then mechanically vibrated for 2 or 3 min. X-ray-diffraction (XRD) patterns of TiO_2_ NPs were obtained at room temperature with a charge-coupled device (CCD) diffractometer (Mercury 3 Versatile CCD Detector; Rigaku Corporation, Tokyo, Japan) using Ni-filtered Cu Kα radiation. The particle sizes of both the powder and the NPs suspended in 0.5% (w/v) HPMC solution after incubation for 24 h (5 mg/mL) were determined using transmission electron microscopy (TEM) (Tecnai G220; FEI Co., Hillsboro, OR, USA) operating at 100 kV. The mean particle size was determined by measuring >100 randomly sampled individual particles. XRD measurements showed that TiO_2_ NPs exhibited an anatase structure with an average grain size of ∼ 6 nm, as calculated from the broadening of the (101) XRD peak of anatase using the Scherrer’s equation. TEM demonstrated that the average size of the particles suspended in HPMC solvent for 24 h was 5–6 nm. The surface area of the sample was 174.8 m^2^/g. The average aggregate or agglomerate size of the nano-TiO_2_ after incubation in 0.5% w/v HPMC solution for 24 h (5 mg/mL) was measured by dynamic light scattering using a Zeta PALS+BI-90 Plus zeta potential analyzer for nanoparticles (Brookhaven Instruments Corp., Holtsville, NY, USA) at a wavelength of 659 nm. The mean hydrodynamic diameter of nano-TiO_2_ in HPMC solvent was 294 nm (range, 208–330 nm) and the zeta potential after 12 and 24 h of incubation was 7.57 and 9.28 mV, respectively [19].

### Ethics Statement

All experiments were approved by the Animal Experimental Committee of the Soochow University (grant no.: 2111270) and performed in accordance with the National Institutes of Health Guidelines for the Care and Use of Laboratory Animals.

### Animals and Treatments

One hundred and twenty female CD-1 (Imprinting Control Region) mice aged 5 weeks with an average body weight (BW) of 23±2 g were purchased from the Animal Center of Soochow University (Jiangsu, China). All mice were housed in stainless steel cages in a ventilated animal facility with a temperature maintained at 24±2°C and relative humidity of 60±10% under a 12-h light/dark cycle. Distilled water and sterilized food were available *ad libitum*. Prior to dosing, the mice were acclimated to the environment for 5 days.

Nano-TiO_2_ powder was dispersed onto the surface of 0.5% w/v HPMC, treated ultrasonically for 30 min, and mechanically vibrated for 5 min. For the experiment, the mice were randomly divided into four groups (n = 30 each), including a control group (treated with 0.5% w/v HPMC) and three experimental groups (treated with 2.5, 5, and 10 mg/kg BW TiO_2_ NPs, respectively). The mice were weighed and then the nano-TiO_2_ suspensions were administered by nasal instillation every day for 90 days. All symptoms and deaths were carefully recorded daily. After the 90-day period, all mice were weighed, anesthetized with ether, and then sacrificed. Blood samples were collected from the eye vein by rapidly removing the eyeball and serum was collected by centrifuging the blood samples at 1,200×g for 10 min. The lungs were quickly removed and placed on ice and then dissected and frozen at −80°C.

### Coefficients of Lung

After weighing the body and lungs, the coefficients of lung mass to BW were calculated as the ratio of lung (wet weight, mg) to BW (g).

### Bronchoalveolar Lavage (BAL) Analysis

After blood collection, the mice were euthanized and the lungs from the control and treated groups were immediately lavaged twice with phosphate buffer saline (PBS). An average of >90% of the total instilled PBS volume was retrieved both times and the amounts did not differ among the groups. The resulting fluid was centrifuged at 400×g for 10 min at 4°C to separate the cells from the supernatant containing various surfactants and enzymes. The cell pellet was used for enumeration of total and differential cell counts as described by AshaRani et al. [20]. Macrophages, lymphocytes, neutrophils, and eosinophils recovered from the BALF were counted using dark field microscopy to assess the extent of phagocytosis. LDH, ALP, and total protein (TP) in the cell-free lavage fluid were analyzed using an automated clinical chemical analyzer (Type 7170A; Hitachi, Ltd., Tokyo, Japan).

### Lung Titanium Content Analysis

The frozen lung tissues were thawed and ∼ 0.1 g samples were weighed, digested, and analyzed for titanium content. Brieﬂy, prior to elemental analysis, the lung tissues were digested overnight with nitric acid (ultrapure grade). After adding 0.5 mL of H_2_O_2_, the mixed solutions were incubated at 160°C in high-pressure reaction containers in an oven until the samples were completely digested. Then, the solutions were incubated at 120°C to remove any remaining nitric acid until the solutions were colorless and clear. Finally, the remaining solutions were diluted to 3 mL with 2% nitric acid. Inductively coupled plasma-mass spectrometry (Thermo Elemental X7; Thermo Electron Co., Waltham, MA, USA) was used to determine the titanium concentration in the samples. Indium (20 ng/mL) was chosen as an internal standard element. The detection limitation of titanium was 0.074 ng/mL and data are expressed as ng/g of fresh tissue.

### Histopathological Analysis

For pathological studies, all histopathological examinations were performed using standard laboratory procedures. The lungs were embedded in paraffin blocks, then sliced (5-µm thickness), and placed on glass slides. After hematoxylin–eosin staining, the stained sections were evaluated by a histopathologist unaware of the treatments using light microscopy (U-III Multi-point Sensor System; Nikon, Tokyo, Japan).

### Observation of Pulmonary Ultrastructure

Lungs were fixed in fresh 0.1 M sodium cacodylate buffer containing 2.5% glutaraldehyde and 2% formaldehyde followed by a 2 h fixation period at 4°C with 1% osmium tetroxide in 50 mM sodium cacodylate (pH 7.2–7.4). Staining was performed overnight with 0.5% aqueous uranyl acetate, then the specimens were dehydrated in a graded series of ethanol (75, 85, 95, and 100%) and embedded in Epon 812 resin. Ultrathin sections were made, contrasted with uranyl acetate and lead citrate, and observed by TEM (model H600; Hitachi, Ltd., Tokyo, Japan). Lung apoptosis was determined based on the changes in nuclear morphology (e.g., chromatin condensation and fragmentation).

### Confocal Raman Microscopy of Lung Sections

Raman analysis of pulmonary glass or TEM slides was performed using backscattering geometry in a confocal configuration at room temperature with an HR-800 Raman microscope system equipped with a 632.817 nm He-Ne laser (JY Co., Fort De, France). Laser power and resolution were approximately 20 mW and 0.3 cm^−1^, respectively, while the integration time was adjusted to 1 s.

### Oxidative Stress Assay

Reactive oxygen species (ROS) (O_2_ **^−^** and H_2_O_2_) production and levels of malondialdehyde (MDA), protein carbonyl (PC), and 8-hydroxy deoxyguanosine (8-OHdG) in the lung tissues were assayed using commercial enzyme-linked immunosorbent assay kits (Nanjing Jiancheng Bioengineering Institute, Jiangsu, China) according to the manufacturer's instructions.

### Microarray and Data Analysis

Gene expression profiles of the lung tissues isolated from control and nano-TiO_2_-treated mice were compared by microarray analysis using Illumina BeadChip technology (Affymetrix, Santa Clara, CA, USA). Total RNA was isolated using the Ambion Illumina RNA Amplification Kit (cat no.1755; Ambion, Inc., Austin, TX, USA) according to the manufacturer’s protocol and stored at −80°C. RNA amplification has become the standard method for preparing RNA samples for array analysis [21]. Total RNA was then submitted to Biostar Genechip, Inc. (Shanghai, China) to analyze RNA quality using a bioanalyzer and complementary RNA (cRNA) was generated and labeled using the one-cycle target labeling method. cRNA from each mouse was hybridized to a single array according to standard Illumina RNA Amplification Kit protocols for all arrays.

Illumina BeadStudio data analysis software (Illumina, Inc., San Diego, CA, USA) was used to analyze the data generated in this study. This program identifies differentially expressed genes and establishes the biological significance based on the Gene Ontology Consortium database (http://www.geneontology.org/GO.doc.html). Differentially expressed genes were identified using the Student’s *t*-test (two-tailed, unpaired) with a threshold of 13.0 to limit the data set to genes up-regulated or down-regulated (DiffScore >13).

### Quantitative Real-time PCR

Expression levels of coagulation factor VII, hydroxymethylglutaryl CoA synthase 2, plasminogen activator - urokinase receptor, tubulin folding cofactor B, and adenosine deaminase *(Ada)* mRNA in the mouse lung tissues were determined using real-time quantitative reverse transcriptase polymerase chain reaction (qRT-PCR) [22]–[24]. Synthesized complimentary DNA was generated by qRT-PCR with primers designed with Primer Express Software (Applied Biosystems, Foster City, CA, USA) according to the software guidelines. PCR primer sequences are available upon request.

### Statistical Analysis

All results are expressed as means ± standard error. Significant differences were examined using the Dunnett’s pair-wise multiple comparison *t*-test using SPSS version 19 software (SPSS, Inc., Chicago, IL, USA). A *p*-value <0.05 was considered statistically significant.

## Results

### BW, Relative Lung Weight, and Titanium Accumulation

Titanium accumulation, BW, and relative lung weight of the mice are listed in Table 1. As shown, an increased nano-TiO_2_ dose led to a gradual decrease in BW, whereas the relative lung weight and titanium content were significantly increased (*p*<0.05), indicating growth inhibition and lung damage in the mice. These findings were confirmed by subsequent pulmonary histological and ultrastructural observations and oxidative stress assays.

**Table 1:** Body weight, relative weight of lung and titanium accumulation in the mouse lung after nasal administration with nano-TiO_2_ for 90 consecutive days.

Index	Nano-TiO_2_ (mg/kg BW)			
	0	2.5	5	10
**Net increase of body weight (g)**	20±1a	16±0.8b	11±0.55c	5±0.25d
**Relative weight of lung (mg/g)**	9.27±0.47a	9.67±0.48a	11.31±0.57b	14.28±0.71c
***Ti content (ng/g tissue)***	Not detected	65±3.25a	113±5.65b	207±10.35c

Letters indicate significant differences between groups (p<0.05). Values represent means ± SE(N = 10).

### Histopathological Lung Evaluation

The histological changes in the lung specimens are shown in Fig. 1. Unexposed lung samples did not exhibit any histological changes (Fig. 1a), while those exposed to increasing nano-TiO_2_ concentrations exhibited severe pathological changes, including infiltration of inflammatory cells, thickening of the pulmonary interstitium, and edema (Fig. 1b–d). In addition, we also observed significant black agglomerates in the lung samples exposed to 10 mg/kg of nano-TiO_2_ (Fig. 1d). Confocal Raman microscopy further showed a characteristic nano-TiO_2_ peak in the black agglomerate (148 cm^−1^), which further confirmed the deposition of nano-TiO_2_ in the lungs (see spectrum B in the Raman insets in Fig. 1d).

**Figure 1:** Histopathology of the lung tissue in ICR mice caused by nasal administration of nano-TiO_2_ for 90 consecutive days. (a) Control group; (b) 2.5 mg/kg BW nano-TiO_2_ group indicates inflammatory cell infiltration (green cycles) and thickening of pulmonary interstitium (green arrows); (c) 5 mg/kg BW nano-TiO_2_ group indicates severs inflammatory cell infiltration (green circles), and great thickening of pulmonary interstitium (green arrows) and pulmonary edema (yellow arrows); (d) 10 mg/kg BW nano-TiO_2_ group indicates severe inflammatory cell infiltration (green arrows) and great thickening of pulmonary interstitium (green arrows), yellow circles show black deposition in the lung. Arrow A spot is a representative cell that not engulfed the nano-TiO_2_, while arrow B spot denotes a representative cell that loaded with nano-TiO_2_. The right panels show the corresponding Raman spectra identifying the specific peak at about 148 cm-1.

### Ultrastructural Changes of the Lung

Changes to the pneumonocytic ultrastructure in the mouse lung samples are presented in Fig. 2. As shown, the untreated mouse pneumonocytes (control) had no abnormal changes (Fig. 2a), whereas the pneumonocytic ultrastructure from the nano-TiO_2_-treated groups indicated a classical morphology characteristic of apoptosis, including mitochondrial swelling, nuclear shrinkage, chromatin condensation, and evacuation of the pneumonocytic lamellar bodies (Fig. 2b–d). In addition, black deposits were observed in the pneumonocytes exposed to 10 mg/kg of nano-TiO_2_ via TEM (Fig. 2d) and Raman signals of nano-TiO_2_ were also exhibited via confocal Raman microscopy (Fig. 2d).

**Figure 2:** Ultrastructure of pneumonocyte in female mice lung caused by nasal administration of nano-TiO2 for 90 consecutive days. (a) Control: chromatin is well distributed, normal lamellar bodies; (b) 2.5 mg/kg BW nano-TiO_2_ indicates a significant shrinkage and chromatin marginalization of the nucleus (yellow arrows), mitochondria swelling(red arrows); (c) 5 mg/kg BW nano-TiO_2_ indicates a significant nucleus pyknosis (green arrows); (d) 10 mg/kg BW nano-TiO_2_ indicate a significant nucleus pyknosis (yellow arrows), mitochondria swelling(red arrows) as well as evacuation of lamellar bodies (green arrows), circles show black deposition. Arrow A spot is a representative cell that not engulfed the nano-TiO_2_, while arrow B spot denotes a representative cell that loaded with nano-TiO_2_. (c) The right panels show the corresponding Raman spectra identifying the specific peak at about 148 cm^−1^.

### Inflammatory Cells and Biochemical Assessments in BALF

To further determine whether long-term nano-TiO_2_ exposure induces lung inflammation, we analyzed inflammatory cell content and biochemical changes in BALF. As shown in Table 2, the numbers of macrophages, lymphocytes, neutrophils, and eosinophils, and LDH, ALP, and TP contents in the nano-TiO_2_-exposed mice showed obvious increases with increasing nano-TiO_2_ dose (*p*<0.05), indicating that nano-TiO_2_ exposure caused severe inflammation and biochemical dysfunction in mice.

**Table 2:** Numbers of inflammatory cells and biochemical changes in BALF of mice after nasal administration with nano-TiO_2_ for 90 consecutive days.

Parameter	Nano-TiO_2_ (mg/kg BW)			
	0	2.5	5	10
**Macrophages (10^4^/per mouse)**	11±0.55a	20±1.0b	36±1.80c	50±2.95d
**Lymphocytes (10^4^/per mouse)**	3±0.15a	6±0.30b	11±0.55c	19±0.95d
**Neutrophils (10^4^/per mouse)**	6±0.31a	14±0.70b	22±1.10c	36±1.80d
**Eosinophils (10^4^/per mouse)**	5±0.25a	10±0.50b	17±0.85c	28±1.40d
**LDH (unit/L)**	582±29a	689±34b	778±39c	986±49d
**ALP (unit/L)**	100±5a	136±7b	188±9c	225±11d
***TP (g/L)***	26.68±1.34a	33.49±1.67b	41.96±2.10c	48.21±2.41d

Letters indicate significant differences between groups (p<0.05). Values represent means ± SE(N = 10).

### Oxidative Stress Analysis

The effects of nano-TiO_2_ on the production of O_2_^−^ and H_2_O_2_ in mouse lung tissues are shown in Table 3. With increasing nano-TiO_2_ dose, the rate of ROS generation in the nano-TiO_2_-exposed groups was significantly elevated (*p*<0.05), suggesting that exposure to nano-TiO_2_ accelerated ROS production in lung tissues.

**Table 3:** Oxidative stress in the mouse lung after nasal administration with nano-TiO_2_ for 90 consecutive days.

Oxidativestress	TiO_2_ NPs (mg/kg BW)			
	0	2.5	5	10
**O_2_^.−^ (nmol/mg** **prot. min)**	23±1.15a	30.27±1.51b	39.18±1.96c	50±2.50d
**H_2_O_2_ (nmol/mg** **prot. min)**	43±2.15a	61.22±3.06b	78.96±3.95c	110±5.50d
**MDA** **(µmol/** **mg prot)**	1.08±0.05a	1.59±0.08b	2.89±0.15c	5.15±0.26d
**Carbonyl** **(µmol/mg** **prot)**	0.54±0.03a	0.98±0.05b	1.85±0.09c	3.04±0.15d
***8-OhdG*** ***(mg/g tissue)***	0.42±0.02a	2.26±0.11b	4.25±0.21c	7.12±0.36d

Letters indicate significant differences between groups (p<0.05). Values represent means ± SE (N = 5).

To further demonstrate the effects of nano-TiO_2_ on ROS generation in mouse lung tissue, the levels of lipid peroxidation (MDA), protein peroxidation (PC), and DNA damage (8-OHdG) were examined. As shown in Table 3, levels of MDA, PC, and 8-OHdG in tissues from the nano-TiO_2_-exposed groups were markedly elevated (*p*<0.05), suggesting that nano-TiO_2_–induced ROS accumulation led to lipid, protein, and DNA peroxidation in the lung.

### Change in Gene Expression Profiles

Treatment with 10 mg/kg BW of nano-TiO_2_ resulted in the most severe pulmonary damage and these tissues were used to detect gene expression profiles to further explore the mechanisms of pulmonary damage induced by nano-TiO_2_. Whole-genome expression profiling using mRNAs from pulmonary tissues of vehicle control groups and those treated with 10 mg/kg BW of nano-TiO_2_ for 90 consecutive days were analyzed with the Illumina Bead Chip. The nano-TiO_2_-treated group was compared with the vehicle control under these criteria: DiffScore ≥13 or ≤ −13 and *p*≤0.05. The results showed that ∼ 1.16% of the total genes (521/45,000 genes with known functions) were significantly changed following nano-TiO_2_ exposure. Of these 521 genes, 361 were up-regulated and 160 were down-regulated. The gene expression profile of the lung tissues from the TiO_2_ NPs-treated mice was classified using the ontology-driven clustering algorithm included with the PANTHER Gene Expression Analysis Software (www.pantherdb.org/). The 521 genes were closely involved in immune responses, inflammatory responses, apoptosis, oxidative stress, metabolic processes, stress responses, signal transduction, cell proliferation, the cytoskeleton, cell differentiation, cell cycling, and so on (Fig. 3), whereas the functions of another 327 genes were unknown. Genes related to immune responses, inflammatory responses, apoptosis, oxidative stress, and the cell cycle are listed in Table 4 (representative genes) and Table S1 (all data).

**Figure 3:** Functional categorization of 521 genes. Genes were functionally classied based on the ontology-driven clustering approach of PANTHER.

**Table 4:** Significant alteration of representative genes after nasal administration of 10 mg/kg BW TiO_2_ NPs for 90 consecutive days.

Symbol		Gene ID	Ontology	DiffScore	Pval
**Immune response**	Defb4	NM_019728	defense response to bacterium	121.33	0
	H2-Oa	NM_008206	regulation of T cell differentiation	−26.34	0
**Inflammatory response**	Chi3l3	NM_009892	inflammatory response	93.12	0
	Alox5ap	NM_009663	leukotriene production involved in inflammatory response	20.37	0
	Il1b	NM_008361	inflammatory response	14.56	0
**Apoptosis**	Pdia2	NM_001081070	apoptosis	73.16	0
	Niacr1	NM_030701	apoptosis	67.22	0
	Ada	NM_007398	negative regulation of thymocyte apoptosis	28.04	0.18
	Sphk2	NM_203280	anti-apoptosis	−13.20	0
	Erbb2	NM_001003817	negative regulation of apoptosis	−14.43	0
**Cell cycle**	Cdkn1a	NM_001111099	cell cycle arrest	15.26	0
	Cdkn1c	NM_001161624	Cell cycle	−15.89	0
**Oxidative stress**	Cryab	NM_009964	oxygen and reactive oxygen species metabolic process	25.36	0
	Alkbh7	NM_025538	oxidoreductase activity	−19.72	0

### qRT-PCR

To verify the accuracy of the microarray analysis, five genes that demonstrated significantly different expression patterns were further evaluated by qRT-PCR due to their association with apoptosis, cell differentiation, blood coagulation, and the cytoskeleton. The qRT-PCR analysis of all five genes displayed expression patterns comparable with the microarray data (i.e., either up- or down-regulation; Table 5).

**Table 5:** Comparison of fold-difference between the control and 90 day 10 mg/kg BW dosage.

Gene	△△Ct	Fold	Microarray
**F7**	−1.786201	3.4490546778	2.458522
**Hmgcs2**	1.163294	0.44649192843	0.523989
**Plaur**	−1.536868	2.9016389168	1.98002
**Tbcb**	−0.004397	1.0030524173	1.562935
**Ada**	−2.280629	4.8588975045	6.867184

## Discussion

The results of the present study indicated that nasal administration of 2.5, 5, and 10 mg/kg of nano-TiO_2_ for 90 consecutive days induced BW reduction, increased relative lung mass, nano-TiO_2_ deposition, (Table 1, Figs 1d, 2d), pulmonary inflammation, thickening of pulmonary interstitium, edema (Fig. 1), and pneumonocytic apoptosis (Fig. 2) in mouse lung tissues coupled with biochemical dysfunction, marked by increased LDH, ALP, and TP levels in the BALF (Table 2), and severe oxidative stress, marked by significant production of O_2_ **^.^** ^−^ and H_2_O_2_, and peroxidation of lipids, proteins, and DNA (Table 3). Furthermore, nano-TiO_2_ exposure significantly increased the influx of inflammatory cells, including macrophages, lymphocytes, neutrophils, and eosinophils, in the BALF (Table 2), further supporting the assertion that nano-TiO_2_ exposure induced pulmonary inflammation. The pulmonary injuries and oxidative stress caused by nano-TiO_2_ exposure may be involved in impaired immune function and antioxidant capacity in mice and, thus, may be associated with altered gene expression in lung tissue. To elucidate the molecular mechanisms of lung damage and identify specific biomarkers induced by nano-TiO_2_ exposure, RNA microarray analysis of mouse lung tissue was performed to establish a global gene expression profile and identify toxicity-response genes in mice following exposure to 10 mg/kg BW of nano-TiO_2_ for 90 consecutive days. Our analysis indicated that the expression levels of 847 genes were significantly changed and 521 of these genes were involved in immune responses, inflammatory responses, apoptosis, oxidative stress, metabolic processes, stress responses, signal transduction, cell proliferation, the cytoskeleton, cell differentiation, and the cell cycle.

In the present study, severe inflammatory responses in the lung tissue occurred due to nano-TiO_2_-induced toxicity (Table 2, Fig. 2). Some studies have demonstrated that ultrafine particle exposure to the respiratory tract can induce pulmonary inflammation [9], [10], [25]–[27]. Latex nanomaterials instilled intratracheally enhanced neutrophilic lung inflammation with pulmonary vascular permeability related to LPS resulting from the activation of innate immune responses [28]. The present study was performed to assess pulmonary immune responses and toxicity in response to nasal administration of nano-TiO_2_ and found that 38 genes (4.49% of 847 genes) involved in immune and inflammatory responses were significantly changed as shown by the microarray data (Table S1). Of these 38 genes, 31 were up-regulated and seven down-regulated. Beta-defensins contribute to the innate and adaptive immune responses in a role as chemoattractants, of which, beta-defensin 4 (Defb4), an antibiotic peptide which is locally regulated by inflammation [29], and the presence of H2-Oa (histocompatibility 2, O region alpha locus) in B cells may serve to focus presentation of antigens internalized by membrane immunoglobulins to increase the specificity of the immune response and avoid reactivity to self antigens [30]. Our data showed that *Defb4* expression was increased by 121.13-fold and *H2-Oa* expression was decreased by 2.69-fold in the nano-TiO_2_-exposed group (Table 4), suggesting that nano-TiO_2_ induced *Defb4* expression and suppressed *H2-Oa* expression, which are both closely related to immune system impairment and inflammation generation (marked by significantly increased levels of macrophages, lymphocytes, neutrophils and eosinophils) in the mouse lung following nano-TiO_2_-induced toxicity. Therefore, we suggest that *Defb4* and *H2-Oa* may be potential biomarkers of nano-TiO_2_ exposure in the lung. In addition, the gene for chitinase 3-like 3 (*Chi3l3*) is characteristically expressed by alternatively activated macrophages. Previous studies have demonstrated innate *Chi3l3* expression in the lungs of infected severe combined immunodeficiency (SCID) mice [31] and eosinophils [32]. Increased Chi3l3 protein expression has been associated with inﬂammatory diseases, in particular with eosinophilic chemotaxis and promotion of cytokine production [33]–[35]. The arachidonate 5-lipoxygenase-activating protein (ALOX5AP) is involved in inﬂammation by mediating the activity of 5-lipoxygenase, which is a regulator of leukotriene biosynthesis, which are pro-inﬂammatory lipid mediators secreted by inﬂammatory cells [36], [37]. IL-1 induces pro- and anti-inﬂammatory response of macrophages. The *IL-1* gene cluster contains three related genes *(IL-1A*, *IL-1B*, and *IL1-RN*), which encode the proinﬂammatory cytokines IL-1α, IL-1β, as well as their endogenous receptor antagonist IL-1ra, respectively [38]. In the current study, nano-TiO_2_ exposure resulted in significantly increased expression of the *Chi3l3*, *Alox5ap*, and *IL1b* genes with the DiffScores of 93.12, 20.37, and 14.56 (Table 4), respectively, indicating a pulmonary inflammatory response, which was closely related to excessive increases of inﬂammatory cells in the lung (Table 2). Taken together, *Chi3l3*, *Alox5ap*, and *Il1b* may be potential biomarkers of nano-TiO_2_-induced pulmonary toxicity.

In the present study, classic morphological characteristics of apoptosis, such as mitochondrial swelling and nuclear chromatin condensation in the pneumonocytes was observed following exposure to 10 mg/kg BW of nano-TiO_2_ (Fig. 1d). To further clarify the apoptotic molecular mechanisms, we analyzed microarray data and found that 31 genes (25 up-regulated and six down-regulated) were altered significantly by exposure to nano-TiO_2_ (Table S1). The expression of several apoptotic mRNAs, including protein disulfide isomerase associated 2, niacin receptor 1, and *Ada* were significantly up-regulated, of which DiffScores were 73.16, 67.22, and 28.04, respectively; whereas sphingosine kinase 2 and v-erb-b2 erythroblastic leukemia viral oncogene homolog 2 were down-regulated with DiffScores of −13.20 and −14.43, respectively (Table 4). As shown in Fig. 4, specifically, the apoptotic pathway analysis showed that nano-TiO_2_ regulated toxicological pathways by increasing the expression of a key factor, Ada, which is an essential enzyme of purine catabolism that is responsible for the hydrolytic deamination of adenosine and 2'-deoxyadenosine to inosine and 2'-deoxyinosine, respectively. These biochemical pathways are essential for maintaining homeostasis, as both Ada substrates have substantial signaling properties. Adenosine engages G protein–coupled receptors on the surface of target cells to evoke a variety of cellular responses, whereas 2'-deoxyadenosine is cytotoxic via mechanisms that interfere with cellular growth and differentiation or the promotion of apoptosis and inflammation [39]. Ada deficiency is a fatal autosomal recessive form of SCID, of which failure to thrive, impaired immune responses, and recurrent infections are characteristics [40], [41]. Adenosine is generated in response to lung hypoxia and injury, and several studies have suggested that this signaling pathway might play an important role in chronic lung diseases, such as asthma and chronic obstructive pulmonary disease [42]–[44]. Therefore, increased *Ada* expression due to nano-TiO_2_ exposure may reduce the accumulation of adenosine and 2'-deoxyadenosine in lung tissue, which in turn can cause cytoprotective or anti-inflammatory responses. *Ada* may be a potential biomarker of lung toxicity caused by nano-TiO_2_ exposure. Since apoptosis is accompanied by altered cell cycle progression, our data suggest that 10 genes involved in the cell cycle were also significantly altered (Fig. 3 and Table S1). Of these 10 genes, seven were up-regulated and three down-regulated. For instance, cyclin-dependent kinase inhibitor (*Cdkn)1a* was increased with a DiffScore of 15.26, whereas *Cdkn1c* was reduced with a DiffScore of −15.89 (Table 4). Among the cell cycle regulatory proteins that are activated following DNA damage, CDKN1A plays essential roles in the DNA damage response by inducing cell cycle arrest, direct inhibition of DNA replication, as well as regulation of fundamental processes, such as apoptosis and transcription [45]. Excessive *Cdkn1a* expression following nano-TiO_2_ exposure may affect DNA damage repair and promote apoptosis in the mouse lung. Since *Cdkn1c* is a cell cycle inhibitor, its role has been largely implicated as a tumor suppressor gene whose loss of function promotes tumor growth and progression [46]. Thus, inhibition of nano-TiO_2_-induced *Cdkn1c* expression is speculated to contribute to apoptotic progression in lung tissue.

**Figure 4:** Ada network pathway obtained from network analysis of differentially expressed genes. Gene Spring software was used to construct and visualize molecular interaction networks.

The present study suggested that nano-TiO_2_ exposure promoted ROS production (such as O_2_^−^ and H_2_O_2_) and led to peroxidation of lipids, proteins, and DNA in mouse lung tissue, indicating oxidative stress, which may be associated with alterations of oxidative stress-related gene expression. Our microarray analysis showed that approximately 22 genes involved in oxidative stress were significantly changed in the nano-TiO_2_-exposed lung (Fig. 3 and Table S1). Of these 22 genes, 11 were up-regulated and 11 down-regulated (Fig. 3 and Table S1). In this study, crystallin-alpha B (*Cryab*) was highly expressed following nano-TiO_2_ exposure, with a DiffScore of 25.36, whereas alkylation repair homolog 7 (*Alkbh7*) was significantly suppressed, with a DiffScore of −19.72 (Table 4). Reportedly, *Cryab* expression in the retina is increased in response to oxidative stress and it has been postulated that this represents a protective mechanism against oxidative stress-induced apoptosis [47]. Elevated *Cryab* expression may increase in response to oxidative stress following nano-TiO_2_-induced pulmonary damage. Alkbh7 is an oxidoreductase, which plays an important role in cardioprotection during ischemia/reperfusion by reducing oxidative stress [48]. In the current study, reduced *Alkbh7* expression induced by nano-TiO_2_ exposure may cause pulmonary peroxisomal disorders and decrease antioxidative capacity or detoxification. Therefore, *Cryab* and *Alkbh7* may be potential biomarkers of nano-TiO_2_–induced pulmonary toxicity.

In regard to the dose selection in this study, we consulted a 1969 study from the World Health Organization, which reported a median lethal dose of TiO_2_ of >12,000 mg/kg BW orally administered to rats. In the present study, we selected 2.5, 5, and 10 mg/kg BW of nano-TiO_2_ and exposed mice to these concentrations every day for 90 days, which was equal to approximately 0.15–0.7 g of nano-TiO_2_ in a human weighing 60–70 kg following such exposure. Although these doses were relatively safe, we recommend using caution for the long-term application of products containing nano-TiO_2_ in humans.

### Conclusion

After exposing mice to nano-TiO_2_ for 90 consecutive days, depositions of nano-TiO_2_ in pulmonary tissues and even in pneumonocytes were observed, which in turn resulted in significant infiltration of inflammatory cells, biochemical dysfunction, oxidative stress, and pneumonocytic apoptosis in mouse lung tissue. The pulmonary injuries following long-term nano-TiO_2_ exposure may be closely associated with significant changes in the expression of genes involved in immune responses, inflammatory responses, apoptosis, oxidative stress, metabolic process, stress responses, signal transduction, cell proliferation, the cytoskeleton, cell differentiation, and cell cycle, specifically, with an increase in *Ada* expression. The obvious elevation in *Ada* expression following nano-TiO_2_ exposure may trigger signaling cascades associated with inflammatory or apoptotic pathways. Therefore, the application of nano-TiO_2_ should be carried out cautiously, especially in humans.

## Supporting Information

Table S1 Genes of known function altered significantly after nasal administration of 10 mg/kg BW TiO_2_ NPs for 90 consecutive days.
(DOC)
